The article "Comparative Analysis of the Effects of the Anti-VEGF Drug and Glucocorticoid by Injection before the End of Vitrectomy for Proliferative Diabetic Retinopathy" was retracted in 2023. Reasons: unreliable results or conclusions; concerns about the data; concerns about the peer review; concerns about the citations.

# Comparative Analysis of the Effects of the Anti-VEGF Drug and Glucocorticoid by Injection before the End of Vitrectomy for Proliferative Diabetic Retinopathy

**DOI:** 10.1155/2021/1285372

**Published:** 2021-10-21

**Authors:** Haijin Zhao, Xueling Li, Xiahai Zhao, Qiongfang Zhang, Wei He, Yanfei Wei, Xueshan Tang

**Affiliations:** ^1^Department of Ophthalmology, Wuzhou Workers' Hospital, Wuzhou, Guangxi 543000, China; ^2^Wuzhou Maternal and Child Health Care Hospital, Wuzhou, Guangxi 543000, China

## Abstract

**Objective:**

To explore the effects of the anti-VEGF drug and glucocorticoid by injection before the end of vitrectomy for proliferative diabetic retinopathy (PDR).

**Methods:**

Eighty PDR patients who underwent vitrectomy in our hospital (July 2020–June 2022) were selected as the research objects and randomized into group A (*n* = 40) and group B (*n* = 40) according to the order of admission. Before the end of surgery, group B was injected with glucocorticoid (triamcinolone acetonide) into the vitreous cavity, and group A was injected with anti-VEGF drug (conbercept). The ophthalmic parameters, incidence of complications, diabetes indexes, and surgical indexes of the two groups were compared.

**Results:**

The best corrected visual acuity (BCVA), central macular thickness (CMT), macular blood flow density and intraocular pressure in group A were remarkably better than those in group B (*P* < 0.001). The incidence of complications (*P* < 0.05) and VEG/F level (*P* < 0.001) in group A were obviously lower than those in group B. There was no significant difference in fasting blood glucose (FBG) and surgical indexes between the two groups (*P* > 0.05).

**Conclusion:**

Conbercept injection before the end of vitrectomy can improve the ophthalmic parameters, reduce the level of VEGF, and lower the possibility of postsurgical complications. Therefore, the low-cost and efficient anti-VEGF drug should be promoted and applied in practice.

## 1. Introduction

Proliferative diabetic retinopathy (PDR) is a common clinical complication of diabetes, with the incidence in diabetes patients as about 2.8%. The pathogenesis is closely related to the overexpression of VEGF and the excessive release of inflammatory factors. The clinical hazards of PDR mainly to lead to blindness and increase the risk of poor prognosis [1]. At present, vitrectomy combined with panretinal laser photocoagulation is commonly used in practice, but patients are prone to bleeding and iatrogenic retinal breaks during surgery, and postsurgical complications such as vitreous rehemorrhage and retinal detachment seriously affect the surgical effect, which may result in patients' irreversible loss of vision [2]. According to its pathological characteristics, perioperative application of anti-VEGF drugs or anti-inflammatory drugs can reduce intraoperative blood loss and the probability of postsurgical complications. Ranibizumab and conbercept are common anti-VEGF drugs, and triamcinolone acetonide is a common anti-inflammatory drug. They all have been used in the study of drug application before vitrectomy, but few studies have applied them before the end of surgery [3, 4]. In particular, there is a lack of specialized research on PDR vitrectomy by using ranibizumab, conbercept, and triamcinolone acetonide. Considering clinical promotion and economic cost, conbercept was chosen as the anti-VEGF drug in this study, and triamcinolone acetonide was chosen as the control drug. This study compared and analyzed the efficacy differences between the above two drugs in PDR patients undergoing vitrectomy. The results are as follows.

The article "Comparative Analysis of the Effects of the Anti-VEGF Drug and Glucocorticoid by Injection before the End of Vitrectomy for Proliferative Diabetic Retinopathy" was retracted in 2023. Reasons: unreliable results or conclusions; concerns about the data; concerns about the peer review; concerns about the citations.

## 2. Materials and Methods

### 2.1. General Data

Eighty PDR patients who underwent vitrectomy in our hospital (July 2020–June 2022) were selected and randomized into group A (*n* = 40) and group B (*n* = 40) according to the order of admission. There was no significant difference in the general data between the two groups (*P* > 0.05) (Table 1). This study was approved by the hospital ethics committee.

### 2.2. Inclusion Criteria

1. Patients or their families fully understood the research and signed the informed consent
2. Patients had a history of diabetes and were diagnosed with PDR by ophthalmic examination [5]
3. Patients presented with vitreous hemorrhage or proliferation by fundus examination and B-ultrasound examination at the PDR stages of IV or V
4. Patients' presurgical blood glucose and blood pressure were well controlled
5. There was no contraindication of vitrectomy
6. The patients' medical data were complete

### 2.3. Exclusion Criteria

1. Patients had mental problems or could not be communicated with
2. Patients suffered from other organic diseases
3. Patients have received similar drug treatment in the past 1 month
4. Patients had surgical contraindications or were unwilling to cooperate
5. Patients were allergic to drugs involved in the study
6. Patients have severe dysfunction of the heart, liver, kidney, lung, and other organs

## 3. Methods

Vitrectomy was performed in both groups. Glucocorticoid (triamcinolone acetonide) was injected into the vitreous cavity before the end of surgery in group B, and anti-VEGF drug (conbercept) was injected in group A. The specific steps were as follows: (1) all patients underwent vitrectomy. The pupil was dilated with compound tropicamide eye drops (Univision Pharmaceutical Co., Ltd.; NMPA approval No. H20066782) and then received retrobulbar anesthesia with 3 ml of lidocaine (Fujian Jinshan Biopharmaceutical Co., Ltd.; NMPA approval No. H35020528) and 3 ml of Ropivacaine (Guangdong Jiabo Pharmaceutical Co., Ltd.; NMPA approval No. H20173194) for minimally invasive 23G vitrectomy. Closed vitrectomy was performed at the pars plana of ciliary body, 4 mm and behind the limbus and behind the three channels. The turbid refractive stroma was removed. The peripheral vitreous body was removed under pressure, the fibroproliferative membrane was removed, and the retina was relaxed. Then, the bleeding was stopped based on the patients' condition, and panretinal laser photocoagulation was performed. The distance between the nasal side and the optic papilla was within 500 um, and the distance between the temporal side and the macular center was within 3000 um. The upper and lower boundaries were within 1–3 spot diameters of the temporal vascular arch, extending beyond the equator. The peripheral retina was pressured to perform photocoagulation to the serrated edge. The total number of laser spots was 2000–2500. The puncture hole was sutured with microbuckwheat thread after removing the casing. If there was lens opacity affecting the surgery, then minimally invasive phacoemulsification and intraocular lens implantation were performed. (2) Glucocorticoid (triamcinolone acetonide): 2 mg of triamcinolone acetonide (Kunming Jida Pharmaceutical Co., Ltd.; NMPA approval No. H53021604) was injected into the vitreous cavity before the end of surgery. (3) Anti-VEGF drug (conbercept): 0.05 ml of conbercept (Chengdu Kanghong Pharmaceutical Co., Ltd.; NMPA approval No. S20130012) was injected into the vitreous cavity before the end of surgery.

The article "Comparative Analysis of the Effects of the Anti-VEGF Drug and Glucocorticoid by Injection before the End of Vitrectomy for Proliferative Diabetic Retinopathy" was retracted in 2023. Reasons: unreliable results or conclusions; concerns about the data; concerns about the peer review; concerns about the citations.

Patients in the two groups were followed up for 3 months after surgery.

### 3.1. Observation Criteria

1. Ophthalmic parameters: it included the best corrected visual acuity (BCVA), central macular thickness (CMT), macular blood flow density, and intraocular pressure. The parameters were compared at 1 week, 1 month, and 3 months after surgery. Among them, the CMT and elevated intraocular pressure were important causes of vision loss, and the larger the value, the worse the surgical effect and poor vision recovery. Macular blood flow density represents the nutritional status of the eye. A higher value is conducive to vision recovery.
2. Incidence of complications: complications included vitreous rehemorrhage, anterior chamber exudation, increased intraocular pressure, lens opacity, and retinal detachment. The number of patients with complications was recorded.
3. Diabetes indexes: it included the VEGF level and fasting blood glucose (FBG). The indexes were compared at 1 week, 1 month, and 3 months after surgery. Specific detection methods: fasting venous blood was collected in the morning, and serum VEGF level and fasting blood glucose were measured by ELISA kit and blood glucose monitor, respectively.
4. Surgical indexes: surgery time, intraoperative bleeding rate, the number of eyes with iatrogenic retinal breaks, and filler application rate of the two groups were compared.

### 3.2. Statistical Processing

In this study, the data were processed by SPSS 20.0 and graphed by GraphPad Prism7 (GraphPad Software, San Diego, USA). Including enumeration data and measurement data, the study used the *X*^2^ test and *t*-test. The differences were statistically significant at *P* < 0.05.

## 4. Results

### 4.1. Comparison of Ophthalmic Parameters

BCVA, CMT, macular blood flow density, and intraocular pressure in group A were remarkably better than those in group B (*P* < 0.001) (Table 2).

### 4.2. Comparison of Incidence of Complications

The incidence of complications in group A was greatly lower than that in group B (*P* < 0.05) (Figure 1).

### 4.3. Comparison of Diabetes Indexes

VEGF level in group A after treatment was remarkably lower than that in group B (*P* < 0.001), and there was no significant difference in FBG between the two groups (*P* > 0.05) (Table 3).

### 4.4. Comparison of Surgical Indexes

There was no significant difference in surgical indexes between the two groups (*P* > 0.05) (Table 4).

## 5. Discussion

Because diabetic patients suffer from hyperglycemia for a long time, the vascular endothelium is damaged, the retinal microvessel is occluded, the transport capacity of oxygen and nutrient reduces, the VEGF transcription increases, the vesicle corpuscle channel is opened, and a new channel for material transport is constructed by protein and fibrinogen. With the reinforcement of blood cells, new blood vessels form. This is the pathogenesis of PDR. For PDR patients who underwent vitrectomy, because of the close connection between neovascularization and retina, it is difficult to completely separate them by vitrectomy alone. Therefore, patients will further suffer from bleeding and iatrogenic retinal breaks for the separation, which leads to high risk of surgery and impairs the optimal therapeutic effect [6–8]. In terms of pathogenesis, neovascularization is closely related to VEGF. Therefore, the perioperative use of anti-VEGF drugs can reduce intraoperative blood loss, reduce the possibility of postoperative vitreous hemorrhage and anterior chamber exudation, and improve the effectiveness of vitrectomy. However, the commonly used ranibizumab in clinical practice is expensive, and the traditional anti-inflammatory triamcinolone acetonide is inclined to generate side effects, although it is cheap. Both cannot meet clinical needs. Therefore, it is vital to find out safe, effective, and inexpensive adjuvant drugs.

The article "Comparative Analysis of the Effects of the Anti-VEGF Drug and Glucocorticoid by Injection before the End of Vitrectomy for Proliferative Diabetic Retinopathy" was retracted in 2023. Reasons: unreliable results or conclusions; concerns about the data; concerns about the peer review; concerns about the citations.

In this study, conbercept is a new generation of anti-VEGF fusion protein developed in China. It can be combined with VEGF, prevent VEGF from signaling reduce the possibility of transcription, and thereby cut down the probability of angiogenesis [9, 10]. At present, there have been studies on the application of conbercept in vitrectomy, but most of them are used for preoperative injection to lighten the impact of intraoperative bleeding on surgical vision, and few studies have applied it before the end of surgery. In this study, conbercept was injected immediately after vitrectomy in order to reduce the dosage and achieve the best therapeutic effect. There was no significant difference in surgical indexes between the two groups (*P* > 0.05), but the incidence of complications in group A was notably lower than that in group B (*P* < 0.05). The results showed that postoperative injection of combretase could still reduce the possibility of postoperative complications such as vitreous rebleeding because combretase could inhibit angiogenesis and reduce retinal inflammatory exudation [11–13]. Thus, patients are not prone to rebleeding due to new blood vessels. It should be noticed that not all PDR patients can be injected with conbercept during the perioperative period. As the retinal vessels are in a wilted state after surgery, ischemia will aggravate in some patients after injection of combretase, which has seriously affected their prognosis. Therefore, whether to inject conbercept depends on the patients' condition in clinical application [14, 15].

This study showed that BCVA, CMT, macular blood flow density, and intraocular pressure in group A after treatment were remarkably better than those in group B (*P* < 0.001). This is related to a lower postsurgical VEGF level in group A. Combretase reduces microvascular permeability, reduces its chance of leakage, and reduces local edema, thereby optimizing CMT. With the improvement of microvascular status, the patient's microcirculation level and macular blood flow density were improved, indicating that the recovery of material transport capacity promoted the recovery of the patient's vision [16–18]. Therefore, for China with 2.5 million PDR patients, conbercept is of high value to be promoted in clinics.

## 6. Conclusion

The injection of conbercept before the end of vitrectomy can improve the ophthalmic parameters of PDR patients, reduce the VEGF level, and lower the possibility of postsurgical complications. Thus, the low-cost and efficient anti-VEGF drug should be popularized in practice.

The article "Comparative Analysis of the Effects of the Anti-VEGF Drug and Glucocorticoid by Injection before the End of Vitrectomy for Proliferative Diabetic Retinopathy" was retracted in 2023. Reasons: unreliable results or conclusions; concerns about the data; concerns about the peer review; concerns about the citations.

## Figures and Tables

**Figure 1:** Comparison of incidence of complications.

**Table 1:** Comparison of patients' general data (*n*, $\bar{x}$ ± *s*).

Group	Group A (*n* = 40)	Group B (*n* = 40)	*t/χ* ^2^	*P*
Gender			0.201	0.654
Male	22	20		
Female	18	20		
Age (years old)				
Range	52–74	53–74		
Average age	61.21 ± 6.20	61.23 ± 6.21	0.014	0.989
Course of diabetes (a)	12.31 ± 3.54	12.36 ± 3.58	0.063	0.950
Fasting blood glucose (mmol)	7.98 ± 0.54	7.99 ± 0.56	0.081	0.935
History of ophthalmopathy (month)	6.21 ± 1.22	6.23 ± 1.23	0.073	0.942
PDR stages			0.251	0.617
IV	28	30		
V	12	10		
Preoperative uncorrected visual acuity	0.44 ± 0.12	0.45 ± 0.11	0.389	0.699
Intraocular pressure (mmHg)	18.98 ± 2.12	18.96 ± 2.23	0.041	0.967
Monthly income (yuan)			0.061	0.805
≥4000	29	28		
<4000	11	12		
Education degree			0.053	0.818
Senior high school degree and below	25	24		
University degree and above	15	16		

**Table 2:** Comparison of ophthalmic parameters (*n*, $\bar{x}$ ± *s*).

Group	Group A (*n* = 40)	Group B (*n* = 40)	*t*	*P*
BCVA (logMAR)				
1 week after surgery	0.29 ± 0.06	0.36 ± 0.08	4.427	≤0.001
1 month after surgery	0.24 ± 0.05	0.30 ± 0.06	4.859	≤0.001
3 months after surgery	0.16 ± 0.03	0.25 ± 0.08	6.662	≤0.001
CMT (*μ*m)				
1 week after surgery	289.98 ± 5.65	300.58 ± 5.89	8.214	≤0.001
1 month after surgery	268.12 ± 5.48	288.68 ± 5.41	16.886	≤0.001
3 months after surgery	245.65 ± 5.44	274.69 ± 5.64	23.439	≤0.001
Macular blood flow density (%)				
1 week after surgery	45.98 ± 1.54	41.41 ± 1.20	14.804	≤0.001
1 month after surgery	46.12 ± 1.22	41.59 ± 1.11	17.370	≤0.001
3 months after surgery	45.14 ± 1.20	41.56 ± 1.24	13.121	≤0.001
Intraocular pressure (mmHg)				
1 week after surgery	17.96 ± 2.12	18.54 ± 2.23	3.894	0.007
1 month after surgery	16.08 ± 2.22	17.05 ± 2.35	3.335	0.009
3 months after surgery	16.54 ± 2.13	17.90 ± 2.25	3.056	0.012

**Table 3:** Comparison of diabetes indexes (*n*, $\bar{x}$ ± *s*).

Group	Group A (*n* = 40)	Group B (*n* = 40)	*t*	*P*
VEGF (*μ*g/L)				
1 week after surgery	400.65 ± 12.56	420.89 ± 12.55	7.210	≤0.001
1 month after surgery	340.89 ± 10.58	378.98 ± 12.44	14.752	≤0.001
3 months after surgery	331.68 ± 12.11	369.65 ± 10.57	14.940	≤0.001
FBG (mmol/L)				
1 week after surgery	7.22 ± 1.20	7.41 ± 1.23	0.699	0.486
1 month after surgery	7.10 ± 1.23	7.20 ± 1.10	0.383	0.703
3 months after surgery	7.00 ± 0.98	7.13 ± 0.99	0.590	0.557

**Table 4:** Comparison of surgical indexes (*n*, $\bar{x}$ ± *s*).

Group	Surgery time (mn)	Intraoperative bleeding rate (%)	Number of eyes with iatrogenic retinal breaks	Filler application rate (%)
Group A	80.12 ± 5.23	20.0 (8/40)	20.0 (8/40)	12.5 (5/40)
Group B	81.44 ± 4.21	30.0 (12/40)	32.5 (13/40)	20.0 (8/40)
*t/χ* ^2^	1.243	1.067	1.614	0.827
*P*	0.217	0.302	0.204	0.363

The article "Comparative Analysis of the Effects of the Anti-VEGF Drug and Glucocorticoid by Injection before the End of Vitrectomy for Proliferative Diabetic Retinopathy" was retracted in 2023. Reasons: unreliable results or conclusions; concerns about the data; concerns about the peer review; concerns about the citations.

## Data Availability

The data used and/or analyzed during the current study are available from all the authors.
